The article "Generation of Human Micro-Doppler Signature Based on Layer-Reduced Deep Convolutional Generative Adversarial Network" was published in 2022. Journal: Comput Intell Neurosci.

# Generation of Human Micro-Doppler Signature Based on Layer-Reduced Deep Convolutional Generative Adversarial Network

**DOI:** 10.1155/2022/7365544

**Published:** 2022-04-12

**Authors:** Mahdi Ostovan, Sadegh Samadi, Alireza Kazemi

**Affiliations:** ^1^Department of Electrical and Electronics Engineering, Shiraz University of Technology, Shiraz 71557-13876, Iran; ^2^Mathematics Department, College of Science, Shiraz University, Shiraz 71348-14336, Iran

## Abstract

Human activity recognition (HAR) using radar micro-Doppler has attracted the attention of researchers in the last decade. Using radar for human activity recognition has been very practical because of its unique advantages. There are several classifiers for the recognition of these activities, all of which require a rich database to produce fine output. Due to the limitations of providing and building a large database, radar micro-Doppler databases are usually limited in number. In this paper, a new method for the generation of radar micro-Doppler of the human body based on the deep convolutional generating adversarial network (DCGAN) is proposed. To generate the database, the required input is also generated by converting the existing motion database to simulated model-based radar data. The simulation results show the success of this method, even on a small amount of data.

## 1. Introduction

Human activity recognition (HAR) has been a popular field of study in the last decade [1–5]. This field of research has attracted the attention of data scientists since the 1980s. HAR is a technology that tries to recognize the activities or movements of the human body through a computer. The purpose of HAR is to recognize the activity of an individual using a series of observations of human behaviors and environmental conditions. In recent decades, various methods have been used to recognize human activities. The methods used can be divided into two main categories: those based on wearable sensors and those based on nonwearable sensors. Wearable sensors require some markers to be attached to a part of the human body for their functionality [6–8]. In applications such as clinical care of the elderly and disabled people, the sensor must be attached to the patient's body and cause inconvenience to them, which is their disadvantage. In contrast, nonwearable sensors such as video surveillance cameras, infrared sensors, and radars do not encounter these problems.

Among the nonwearable sensors, radar has shown its application as well. The advantages of using radar for HAR are as follows:

1. Radar is resistant to light and weather conditions. Therefore, it can be used in environments with adverse conditions.
2. The radar sensor maintains the visual privacy of people. Because instead of extracting the visual form of the body, it uses target-modulated return signals that contain valuable information about the range and speed of the moving target.
3. Radar can detect humans even through walls, which makes it useful in more scenarios.
4. Radar does not need to attach a marker to a human target for its operation. This makes it more user-friendly.

The human body is a nonrigid target. In addition to the translational motion of the whole body, the locomotion of the body parts is also significant. The instantaneous distance of the body parts to the radar changes with micromotions, and it induces the effects of micro-Doppler on the echo signal [9]. The radar micro-Doppler signature carries unique and valuable information about moving targets, which has received much attention in the classification, recognition, and identification of human targets.

An issue that has always been a major concern in machine learning-based classification problems is how to prepare a standard, large, and diverse enough database. In camera-based classification methods, the camera sensor is publicly available, many images and videos of people's daily lives and activities are recorded, and usually many databases are available for these sensors [10, 11]. However, radar is not a typical sensor and is accessible only to certain people. So, the radar databases are very limited and sometimes not available due to some security issues. Lack of sufficient volunteer humans, costly radar data recording tests, long preparation time of the test environment, and such issues make providing radar database very difficult and rather challenging. Therefore, the challenge we are dealing with is the collection of diverse and appropriate data. Attempts have been made to increase the data in a way other than direct testing.

One of the methods used in various literature is the computer simulation method. In this method, data are generated statistically from scratch using human kinematic models. The most famous kinematic model of the body is the Boulic gait model [12]. In this model, given a limited number of body parameters such as height and thigh length, the human gait model can be simulated. This method has been validated many times, including [13, 14]. It has been used as a reference for walking simulation. Although this method can generate an unlimited amount of data for deep network training, it is limited to the walking model and can also be used for running with little modification, but it is not applicable for other activities, such as crawling and sitting. In [15], a method for simulating micro-Doppler signatures of running and crawling in addition to walking activity has been proposed using virtual reality animation. However, the diversity of models is not significant.

The most widely used method is using the Kinect sensor for Microsoft's Xbox game console [16, 17]. This camera has two optical sensors and an IR sensor. By integrating the data from these three cameras, it has been able to measure the depth and instantaneous location of the joints in the human body with an accuracy of better than 1 cm. Thus, a model provides a simplified point of the human body at about 18 to 30 frames per second (depending on software and hardware conditions) in 3D space.

The locations of these body joints can be used to simulate the radar echo signal [9, 18], which is a widely used method that is close to reality. In this method, a 17-point model equivalent to the Boulic model is extracted from the joints of the test object. Each limb is then assigned a simple geometric shape. All body parts (except the head) are assigned an ellipse, and a sphere is assigned to the head. By calculating the RCS of each limb according to physical relations, the radar echo can be simulated. After that, the echo in the time domain is transformed to the time-frequency domain by a transform such as the STFT. This method has also proven its efficiency and closeness to reality. The use of the Kinect will be limited due to the very short operational range (less than 2 meters) and the missed detection of some limbs, such as the legs [17].

Another method to solve the problem of data shortages is using a method known as transfer learning. In this technique, a few network layers that have already been trained on a large database are used in the designed network. The initial database should be somewhat close to our desired task. Usually, the primary layers of the deep grid are responsible for extracting general and basic features, and therefore, a series of general features can be extracted regardless of the input contents. In contrast to deeper layers, they extract minor features. So, if we maintain the primary layers of a deep network trained with a large database and retrain and replace the deep layers with a database of related data, which is called “fine-tuning,” then we will be able to achieve the required accuracy with a small amount of data. References [19–25] have used this method to improve classification with a small amount of data. However, it is often difficult to find a database close enough to the radar micro-Doppler problem. Although using heterogeneous and irrelevant databases can train the primary layers of the network, they can also take us away from our destination. Radar micro-Doppler images are composed of several lines and curves and using natural pictures to train the transferred network will produce unpromising results as they contain completely different content.

A new method that has recently been discussed to produce a realistic image [26–29] is the use of generating adversarial networks, or GAN for short. The faces in Figure 1 are simulated using the DCGAN network trained with the CelebA database [30]. This database contains more than 200,000 faces of Hollywood actors and singers around the world. The faces in Figure 1 do not exist in the real world, but they look like real faces, and that shows the power of GAN.

Due to the weakness of the mentioned methods and the novelty and power of GAN networks in making realistic images, in this paper, we have proposed a new method for generating human body radar micro-Doppler based on the deep convolutional generative adversarial network (DCGAN) using a simulated database. The structure of the paper is as follows: Section 2 describes how to generate our database.  Section 3 provides an overview of GANs.  Section 4 introduces the proposed GAN network.  Section 5 presents the results of the simulations. Finally, Section 6 is devoted to the discussion and conclusion.

## 2. Database Preparation

We used the MoCap motion capture database of CMU [31] to simulate radar echo. In this relatively rich database, various activities have been performed by volunteers, and their body locomotions, have been recorded by very accurate multi-modal motion sensors. They are a combination of cameras and inertial sensors like gyroscopes and accelerometers. We have focused only on walking activities. The data recorded in the MoCap output related to the bodies of walking people was first extracted in the point model. The number of points is up to 40, but we used only 17 points, according to [9].  Figure 2 shows a frame of the 17-point body model extracted from the CMU database and simulated by the routine of [9].

According to this method, an ellipsoid is assigned to each limb except for the head, which is spherical. These geometric shapes move according to the instant locations of body joints. The temporal coordinates of the body parts are extracted from data provided by [32] in the form of [*x*(t), *y*(*t*), *z*(*t*)]^T^. By micromotion of these shapes, radar echo data is simulated. The signal at this stage is generated in the range-time domain. Finally, the simulated echo signal is transformed into the time-frequency domain. We used the FSST transform introduced in [33], whose time-frequency resolution is better than STFT. A synchro-squeezing process is applied to the time-frequency domain to make it sharper along the frequency axis. A comparison of FSST and STFT is performed in [34] and is depicted in Figure 3. As we can see, the resolution of FSST is better than that of STFT.

After transforming into the T-F domain, the echo signal of each trial is stored as an image like Figure 3(a). In this way, the initial data were generated to enter the DCGAN.

## 3. Generative Adversarial Networks

The GAN network, first introduced in [26], implements the game theory method by training two different networks, one as a generator and the other as a discriminator. The generator network is represented by the *G* function and is parameterized by *θ*_*g*_ and initialized with an input noise vector *z*, which consists of samples of a normal distribution. (*P*_*noise*_ (*z*)) and its output is *Î*.

The discriminator network is a convolutional neural network (CNN) represented by the *D* function and is parameterized by *θ*_*d*_. Its input is a real image *I* or a fake image *Î,* and its output is a number between 0 and 1 that indicates the probability that the input is real or fake. Training of the GAN includes a minimax game [35] in which the generator tries to fool the discriminator so that it cannot recognize fake images from real ones. Meanwhile, the discriminator is trying to identify them correctly.

*D* is trained to maximize the probability of assigning the correct label to both training samples and generated samples of *G*. At the same time, *G* is trained to minimize the log(1 − *D*(*G*(*z*)), in other words, *D* and *G* play the minimax game with the value of the *V*(*G*, *D*) as given inthe following equation:

(1) $$\begin{array}{c} \underset{G}{\text{min}}\underset{D}{\text{max}}V\left(D,G\right)=E_{x∼p_{\text{data}}\left(x\right)}\left[\log\;D\left(x\right)\right]+E_{z∼p_{z}\left(z\right)}\left[\log\left(1-D\left(G\left(z\right)\right)\right)\right], \end{array}$$

where *P*_*g*_ is the probability distribution of *G* on set *x*, *G*(*z*, *θ*_*g*_) is a differentiable function with parameters *θ*_*g*_, and *D* (*x*;*θ*_*d*_) is a differentiable function with parameters *θ*_*d*_.

After several training iterations, if *G* and *D* have enough training capacity, they will reach a final point in which the training error does not decrease further. At this point, *P*_*g*_ = *p*_*data*_ and the discriminator does not have enough power to discriminate between two distributions. Now network *G* is ready to generate fake samples with maximum similarity to real samples and with the same statistical distribution. A basic GAN block diagram is depicted in Figure 4.

## 4. Proposed DCGAN Network

In [29], a kind of convolutional GAN network called DCGAN is used to produce realistic images. Due to the success of GAN networks in various studies, in this paper, we have used a kind of DCGAN to generate the micro-Doppler signal of the walking human in the T-F domain. The original DCGAN was trained on the LSUN database [36], Imagenet-1k [37], and CelebA [30]. The contents of these databases are about natural scenes, which have many details. Our proposed discriminator network structure has only four convolutional layers. The purposes for reducing the convolutional layers are as follows:

1. The network is trained to generate the micro-Doppler signal in the time-frequency domain, which is composed of some periodic curves, and unlike natural images, it does not have much detailed information.
2. Computational load could be reduced by the simplification of network structure.

The architecture of the generator network is shown in Figure 5 and the discriminator network in Figure 6.

The generator network is composed of five transposed convolutional layers followed by a batch normalization layer for the stability of training progress and an activation layer of type rectified linear unit (ReLU).  Table 1 lists the parameters of the generator network.

The parameters of discriminator network are listed in Table 2.

These two networks are trained simultaneously on our database using the Adam optimization method. The output images from the simulated database described in Section 2 will enter into the discriminator network of Figure 5. Simultaneously, noise with a length of 100 samples enters the generator network of Figure 6. As a result of the training described previously, the statistics of the data generated by the generator network gradually approach the statistics of the samples within the database.

## 5. Simulation Results

In this section, we have reported the simulation results of generating curves by the proposed DCGAN network.

### 5.1. Simulation Platform

Training of deep neural networks usually encounters challenges. The first challenge is the high computational load, which forces us to use powerful processing platforms. In the simulations presented in this paper, due to the modifications that are performed on the network structure and the small number of input trials in the database, a CPU-based platform has been used.

### 5.2. Training Options

Hyperparameters of training are selected as in Table 3.

According to Table 1, the number of trials in the simulated database is only 81. However, the output is very close to reality and promising. In the simulation process, as the training epochs increase, the input noise gradually proceeds to true form. Figures 7(a)to 7(c) show the network output at different stages of training. As the training progresses, the output gets closer to the expected shape.  Figure 7(d) shows a comparison of one of the real samples of the database, which is very close to output 5c.

### 5.3. Evaluation

Because the output of the DCGAN network is random, it cannot be evaluated in terms of traditional image comparison criteria such as PSNR because the ground truth could not exist. However, it is important to note that the matching of generated data statistics and database statistics is the optimization criterion of the adversarial learning process, and it converges when these statistics are matched. Thus, the adversarial network ensures that the output image statistics and the database images are the same, which can be considered a quantitative evaluation and a complement to the visual evaluation.

The histogram of an image is a demonstration of the intensity levels and can represent the distribution of these intensities. To show that the trained network is able to generate good fake results, we have compared the average histogram of some samples in the database with some generated samples.  Figure 8, shows the results. The result demonstrates the similarity of statistics.

As a second metric for similarity measurement of the real and fake images, we used the structural similarity index measure (SSIM) [38]. SSIM is a good metric to show perception and saliency-based errors. Therefore, we can conclude that SSIM could be comparatively a better metric than mean square error (MSE) and PSNR metrics from a human visual perspective. The term structural information emphasizes pixels of the image that are strongly interdependent or pixels that are spatially interconnected. Highly dependent image pixels provide more valuable information than visual objects in the image domain [39]. The SSIM metric is an index in [0,1] with 0 indicating no similarity and one indicating maximum similarity.

For comparison, we have calculated SSIM between 100 generated images and every image in the database and averaged them, as shown in Figure 9. The consequent average value is about 0.94, which represents a very high similarity between generated images and real samples.

## 6. Conclusions

In this paper, a new method based on the use of the DCGAN for the production of micro-Doppler of the human body is presented. The database required for this work was generated using a computer simulation of the radar echo signal based on the 17-point body model while considering the system parameters of a typical radar. Motion data of 17 body parts and their kinematics are taken from the MoCap database of CMU University. The production database for the input of the proposed method has only 81 members, but the result is very promising. In the future, we will seek to increase the database and train this network with more diverse data. The results of this work provide a valuable tool for future research in the field of classification of human activities based on radar micro-Doppler.

## Figures and Tables

**Figure 1:** Simulated faces with DCGAN [29].

**Figure 2:** 17-point simulated body.

**Figure 3:** Comparison of (a) FSST and (b)–(f) STFT with different window lengths [32].

**Figure 4:** Block diagram of a basic generative adversarial network.

**Figure 5:** Generator network.

**Figure 6:** Discriminator network.

**Figure 7:** (a) Input noise to GAN. (b) Output after 150 epochs. (c) Output after 1000 epochs. (d) A real sample.

**Figure 8:** Comparison of the histograms of the real and generated samples.

**Figure 9:** SSIM calculated over generated samples and real samples.

**Table 1:** Parameters of generator network.

Row	Layer name	Layer type	Attribute
1	Input noise	Image input	1 × 1 × 100 noise vector
2	TConv 1	Transposed convolutional	512 tconv filters of size 4 × 4 with stride [2, 2] and cropping [0, 0]
3	BN1	Batch normalization	—
4	ReLU 1	ReLU	—
5	TConv 2	Transposed convolutional	512 tconv filters of size 4 × 4 with stride [2, 2] and cropping [0, 0]
6	BN2	Batch normalization	—
7	ReLU 2	ReLU	—
8	TConv 3	Transposed convolutional	512 tconv filters of size 4 × 4 with stride [2, 2] and cropping [0, 0]
9	BN3	Batch normalization	—
10	ReLU 3	ReLU	—
11	TConv 4	Transposed convolutional	512 tconv filters of size 4 × 4 with stride [2, 2] and cropping [0, 0]
12	BN4	Batch normalization	—
13	ReLU 4	ReLU	—
14	TConv 4	Transposed convolutional	512 tconv filters of size 4 × 4 with stride [2, 2] and cropping [0, 0]
15	tanh	Hyperbolic tangent	—

**Table 2:** Parameters of discriminator network.

Row	Layer name	Layer type	Attribute
1	Input image	Image input	64 × 64 × 3 images
2	Conv 1	Convolutional	64 conv filters of size 4 × 4 with stride [2, 2] and padding [1, 1]
3	Leaky ReLU 1	Leaky ReLU	Scale of 0.2
4	Conv 2	Convolutional	128 conv filters of size 4 × 4 with stride [2, 2] and padding [1, 1]
5	BN2	Batch normalization	—
6	Leaky ReLU 2	Leaky ReLU	Scale of 0.2
7	Conv 3	Convolutional	256 conv filters of size 4 × 4 with stride [2, 2] and padding [1, 1]
8	BN3	Batch normalization	—
9	Leaky ReLU 3	Leaky ReLU	Scale of 0.2
10	Conv 4	Convolutional	1 conv filter of size 8 × 8 with stride [1, 1] and padding [0, 0]

**Table 3:** Training hyperparameters.

Parameter	Value
Epoch	1000
Mini batch size	8
Generator learning rate	2 × 10^−4^
Discriminator learning rate	1 × 10^−4^
Gradient decay factor	0.5
Squared gradient decay factor	0.999
Number of samples	81

## Data Availability

The data we have used is given from the publicly available online Carnegie Mellon University (CMU) motion capture database [32], [online] available from https://mocap.cs.cmu.edu/.
